# Back Propagation Neural Network-Based Ultrasound Image for Diagnosis of Cartilage Lesions in Knee Osteoarthritis

**DOI:** 10.1155/2021/2584291

**Published:** 2021-07-30

**Authors:** Xiaoming Zhao, Wei Gong, Xing Li, Weibing Yang, Dengfeng Yang, Zhiguo Liu

**Affiliations:** ^1^Department of Orthopaedics, Baoji Central Hospital of Shaanxi Province, Baoji 721008, Shaanxi, China; ^2^Department of Bone and Joint Trauma, Hanzhong City Center Hospital, Hanzhong 713000, Shaanxi, China

## Abstract

**Objective:**

To explore the application value of ultrasound image based on back propagation (BP) neural network algorithm in knee osteoarthritis (KOA) and evaluate the application effect and value of ultrasound image technology based on the BP neural network in the diagnosis of knee osteoarthritis cartilage lesions, 98 patients who were admitted to our hospital were diagnosed with KOA and had undergone arthroscopic soft tissue examinations were randomly selected. According to whether image processing was performed, the ultrasound images of all patients were divided into two groups. The control group was image before processing, and the experimental group was image after processing optimization. The consistency of the inspection results of the ultrasound images before and after the processing with the arthroscopy results was compared. The results showed that the staging accuracy of the control group was 68.3% and that of the experimental group was 76.9%. The accuracy of staging cartilage degeneration of the experimental group was higher than that of the control group, and the difference was not remarkable (*P* > 0.05). The kappa coefficient of the experimental group was 0.61, and that of the control group was 0.40. The kappa coefficient of the experimental group was higher than that of the control group, and the difference was significant (*P* < 0.05).

**Conclusion:**

The inspection effect of the ultrasound image processed by the BP neural network was superior to that of the conventional ultrasound image. It reflected the good adoption prospect of neural networks in image processing.

## 1. Introduction

Knee osteoarthritis (KOA) is a common joint degenerative disease in clinical orthopedic diseases, also known as osteoarthritis, degenerative arthritis, etc. [1]. Most of the people with high incidence of KOA are the elderly. Therefore, with the aging of China's population, the disease also gradually presents an upward trend [2]. The general clinical manifestations of KOA are knee pain and limitation of movement, but it often causes joint soft tissue lesions such as cartilage, subchondral bone, synovial capsule of the joint, and knee osteoarticular ligament in severe cases. Then, along with the development of pathological changes, cartilage tissue damage, bone spurs, and even joint deformation can lead to bone and joint failure [3–5], which will bring great inconvenience to the life of patients. At present, the main treatment for knee cartilage lesions is conservative treatment, which is targeted at the early stage of knee cartilage lesions. Arthroscopic therapy may be appropriate for patients with stage II lesions according to the condition of the disease. Surgical treatment is recommended for patients with stage III to moderate lesion stage [6–8]. Accurate diagnosis is essential in order to adopt reasonable and appropriate treatment methods and ensure the treatment effect. At present, the diagnosis of KOA joint disease is mainly based on the results of imaging techniques, including X-ray, CT, MRI, and ultrasound. However, X-ray and CT have great limitations in the display of soft tissue around the joint, which cannot be well displayed. Although MRI can display the soft tissue lesions around the joint, there are still many inconveniences [4, 9, 10]. Therefore, ultrasonic testing has been favored by more people due to its high-resolution display characteristics, noninvasiveness, safety and simple operation mode, and easy-to-accept test price [11]. With the continuous adoption of this technique in clinical practice, its accuracy in the examination of KOA disease and peripheral soft tissue lesions caused by this disease has become a hot spot in clinical research.

At present, ultrasound imaging technology is mainly used for the detection of Doppler ultrasound imaging, by showing the patient's disease location to the doctor in the form of black-and-white image to diagnose the disease. With the rapid development of artificial intelligence (AI) technology, its algorithm has been widely used in medical image processing. The principle of this technology is extracting the feature map of the original image and comparing it with the expert's to make a detection diagnosis [12]. AI algorithms include a kind of neural network calculation that has been used in various industries. Among them, the back propagation (BP) feed forward neural network is a kind of AI learning algorithm, which is widely used at this stage. It can well process images and has good adoption value in forecasting [13]. The principle of the BP neural network is as follows. Firstly, the corresponding network connection weight is obtained through the given training samples. Secondly, the input samples to be processed are taken to obtain the corresponding output samples. When the process is completed, the weight will not be changed. To put it simply, the training process of neural network algorithm for image processing is actually a process of obtaining network weights, and the methods to obtain them are mainly the back propagation of error and the speediest gradient method [14].

In this study, it used the BP neural network algorithm to optimize the ultrasound image of KOA cartilage lesions for the diagnosis of the disease and compare with the results of conventional ultrasound image examination, so as to evaluate the application effect and value of ultrasound image technology based on the BP neural network in the diagnosis of knee osteoarthritis cartilage lesions. It aimed to study more effective and feasible detection techniques for clinical diagnosis and treatment of KOA patients.

## 2. Methods

### 2.1. Research Objects

A total of 98 patients with KOA who were admitted to our hospital from October 2018 to March 2020 and had undergone arthroscopic soft tissue examination by arthroscopy were randomly selected in this study. Among them, 42 male patients and 56 female patients ranged in age from 50 to 78 years old, with an average age of (64.3 ± 7.9) years old. All patients had completed ultrasound diagnosis at admission, with complete arthroscopic results and general clinical data. The ultrasound images of all patients were processed and optimized by the BP neural network algorithm, and the consistency between the ultrasound images and arthroscopy results before and after treatment was compared. Ultrasound images of all patients were divided into two groups according to whether image processing was performed. The group before processing was set as the control group, and the group after optimized processing was set as the experimental group. This study had been approved by the medical ethics committee of our hospital. The patients and their families were informed of the study and signed the informed consent.

Inclusion criteria: (a) according to the diagnostic criteria for KOA prescribed by the American Rheumatology Association (ACR) in 2001 [15], as shown in Figure 1, patients with knee pain were diagnosed as KOA if they had five of the following nine items. (b) All patients were over 50 years old (inclusive). (c) None of the patients had undergone surgical treatment for KOA.

Exclusion criteria: (a) patients complicated with severe cardiovascular and cerebrovascular diseases and severe dysfunction of the liver, kidney, and hematopoietic system. (b) Patients with KOA lesions due to other causes and cartilage lesions around joints.

### 2.2. Experimental Methods

#### 2.2.1. Inspection Method

First, high-frequency ultrasound examination was performed on all patients. All patients were scanned using the same machine and equipment, and all the examination process were carried out by the same experienced, skilled, and accurate imaging doctor. The linear array probe was used for the ultrasonic equipment, and the probe frequency was set at 10 MHz.  Figure 2 showed the specific operation. Then, arthroscopy was performed on the patients who needed it. The procedure must be performed by two experienced orthopedic surgeons, and all patients were treated with a unified arthroscopic device to avoid greater individual differences. The degeneration of knee cartilage was staged according to the staging criteria in Table 1. The process of reviewing the ultrasound images was carried out by two highly qualified imaging doctors. The state of the cartilage surface around the joint, the echo state of the ultrasonic image inside the cartilage, and the morphological changes of part of the cartilage were mainly evaluated, and the thickness of the cartilage was measured. According to Table 2, lesions were staged. When the result is different, the final result should be agreed through discussion and consultation.

#### 2.2.2. Ultrasonic Image Based on the BP Neural Network Algorithm

BP neural network algorithm was adopted to denoise and optimize the image under the ultrasonic image technology. The algorithm process is as follows.

First of all, the speckle noise in the ultrasonic image was studied. According to the study, if the particles scattered in the human tissues are sufficient and evenly distributed, the distribution of speckle noise in ultrasonic images conforms to Rayleigh distribution and is expressed by the multiplicative model in the following equation:

(1) $$\begin{array}{c} Q=we. \end{array}$$

*Q* in equation (1) represents the undenoised image disturbed by noise *e*, and *w* is the original undisturbed image. If the noise distribution conforms to Rayleigh distribution, the following equation is obtained:

(2) $$\begin{array}{c} R=f\left[\sum tQ\right]. \end{array}$$

In equation (2), *f* is a nonlinear function, which is relatively complex; *t* is the nonlinear coefficient; and *R* is the result of nonlinear transformation after the weighted sum of gray values of all pixels in the noisy image *Q*.

The processing of the BP neural network is the forward signal transmission of the original image-reverse transmission error-continuous training and correction-inspection effect. The BP network includes input layer, hidden layer, and input layer. During training, the output relationship of the BP neural network is represented by equation (3), where *W*_*i*_, *X*_*i*_, *O*_*i*_, and *y* represent the weight, input value, bias, and output value of the *i*th neuron in the hidden layer, respectively.

(3) $$\begin{array}{c} y=\sum_{i=0}^{T-1}w_{i}x_{i}+o_{i}. \end{array}$$

The error function calculation method in the back propagation process is shown in the following equation, where *a*_*j*_ is the output result of node *j*.

(4) $$\begin{array}{c} P\left(w,o\right)=\frac{1}{2}\sum_{j=0}^{s-1}{\left(a_{j}-d_{j}\right)}^{2}. \end{array}$$

The optimization algorithm of the BP neural network often uses the gradient descent method, as shown in equation (5), where *β*_*i+1*_ is the weight after optimization, *β*_*i*_ is the weight before optimization, *α* is the learning probability, and *χJ*(*β*)/*χβ*_*i*_ is the gradient in the weight direction.

(5) $$\begin{array}{c} \beta_{i+1}=\beta_{i}-\alpha \frac{\chi J\left(\beta \right)}{\chi \beta_{i}}. \end{array}$$

At this time, the BP neural network obtains the relational expression of the function, and the training is completed. The denoising effect is evaluated regarding peak signal-to-noise ratio, which is expressed by the following equation:

(6) $$\begin{array}{c} F=101g\left[\frac{\max{\left(h\right)}^{2}}{\mathrm{MSE}}\right]. \end{array}$$

In equation (6), *h* is the ultrasonic image after denoising and MSE is mean square error, which is calculated in equation (7), where *h*_0_ is the original unprocessed ultrasound image and *M* is the ultrasound image number:

(7) $$\begin{array}{c} \mathrm{MSE}=\frac{\sqrt{{\sum_{i=1}^{M}\left(h-h_{0}\right)}^{2}}}{M}. \end{array}$$

The before and after comparison of the optimized ultrasound image processed by the BP neural network algorithm is shown in Figure 3.

### 2.3. Statistical Methods

SPSS 22.0 was employed for data entry, sorting, and statistical analysis. The comparison of count data was performed by *χ*^2^ test, while the comparison of measurement data was performed by *t*-test. Multiple sample means were compared using analysis of variance. The LSD method was used when the variance was uniform, and the Dunnett T3 method was used when the variance was uneven. *P* < 0.05 was statistically different. The kappa test was performed on the consistency between the staging results shown in the two groups of ultrasound images and those seen under arthroscopy. When kappa > 0.75, the consistency between the two was strong. When 0.4 ≤ kappa < 0.75, the consistency between the two was general. When kappa < 0.4, the consistency between the two was poor.

## 3. Results

### 3.1. Staging Results of Cartilage Lesions under Arthroscopy

98 patients were examined for cartilage lesions on a total of 490 articular surfaces under arthroscopic surgery. Among them, the cartilage of 206 articular surfaces was normal and uninvolved and caused disease. The cartilage of the remaining 284 articular surfaces had different degrees of disease, with a total of 320. Among them, 56 were in stage I, 85 were in stage II, 94 were in stage III, and 85 were in stage IV. The staging results of different detection parts are summarized in Table 3.  Figure 4 shows the performance of different stages under arthroscopy. It was obvious that the pathological differences of the cartilage around the joints in each stage can be observed.

### 3.2. The Staging Results of Cartilage Lesions under Ultrasound Imaging in the Control Group

Among cartilage lesions on 490 articular surfaces of 98 patients in the staging results of the ultrasound image of the control group, the echo distribution of the ultrasound image of cartilage with 242 articular surfaces was a normal high-low-high distribution. The cartilage of the remaining 248 articular surfaces all had different degrees of lesions, with a total of 284 lesions. Among them, 38 were in stage I, 99 were in stage II, 83 were in stage III, and 64 were in stage IV. The staging results of different detection sites are summarized in Table 4.  Figure 5 shows the ultrasound imaging manifestations of different stages of the control group. There were certain differences in the pathological changes of the cartilage around the joints in each stage.

### 3.3. The Results of Staging of Cartilage Lesions under Ultrasound Imaging in the Experimental Group

Among cartilage lesions on 490 joint surfaces of 98 patients in the staging results of the ultrasound image of the experimental group, the echo distribution of the ultrasound image of cartilage with 231 articular surfaces was normal. The cartilage of the remaining 269 articular surfaces had different degrees of lesions, with a total of 307 lesions. Among them, 44 were in stage I, 87 were in stage II, 87 were in stage III, and 89 were in stage IV. The staging results of different detection sites are summarized in Table 5.  Figure 6 shows the ultrasound image manifestations of different stages in the experimental group. There were certain differences in the lesions of the cartilage around the joints in each stage.

### 3.4. Comparison of Consistency between the Staging Results of the Two Groups of Ultrasound Images and the Results under Arthroscopy

The examination results of the two sets of ultrasound images of the cartilage lesions around the KOA of all patients were compared with the results observed under arthroscopy. There were 335 cartilage degenerations that were accurately detected by the ultrasound image of the control group, and the staging accuracy of the inspection results was 68.3%. In the experimental group, 377 cartilage degenerations were detected, and the staging accuracy of the inspection results was 76.9%. The accuracy of staging of cartilage degeneration in the experimental group was higher than that in the control group, but the difference was not remarkable (*P* > 0.05). Moreover, the kappa coefficient of the ultrasound image staging and arthroscopic staging results of the experimental group was 0.61, while the kappa coefficient of the control group and arthroscopic staging was 0.40. The kappa coefficient of the two groups indicated that they were generally consistent with the arthroscopic staging results, but the kappa coefficient of the experimental group was higher than that of the control group, with considerable difference (*P* < 0.05), as presented in Figure 7.

## 4. Discussion

The progression of KOA disease is very likely to cause degenerative lesions of the cartilage around the knee joint. Patients will feel the pain of the knee joint, flexion, and extension, which even bring difficulties in walking, seriously affecting the patient's daily life. Therefore, timely and effective diagnosis is necessary for the control of cartilage involvement in patients with KOA. In order for the treatment to be effective, symptomatic treatment is necessary. The accuracy of examination of the degree of knee cartilage degeneration has an effective guiding significance for doctors to make a reasonable clinical treatment plan. There are a variety of detection methods for KOA disease, including MRI, X-ray, CT, and ultrasound, but all of them have certain adoption limitations. Ultrasound diagnosis has been welcomed by its effect on the adoption of research analysis which has been analyzed by a lot of researchers and clinicians for its excellent characteristics such as no radiation, low cost, short examination time, and simple operation, especially for the diagnosis of osteoarthritis. Researchers studied the effectiveness of ultrasound in the detection of cartilage lesions in the knee. It was found that when the knee joint was in complete flexion, ultrasound examination could clearly show the tissue structure of the cartilage around the joint, including the trochlea, femur, and medial and lateral condyle. Other researchers proposed that when the knee flexion angle was maximized, the articular surface of the patella pulley was fully exposed. The blocked range of the medial and lateral condyles of the femur can also be reduced, so that it can observe the cartilage lesions on the articular surface of the femur more completely [16]. In this study, the knee flexion of the two aspects was observed, and the results were basically the same, except that the femoral articular surface could not be fully exposed due to various obstructions. In addition, it was found through studies that ultrasound imaging can show significant differences in the degree of cartilage degeneration, which can be regarded as an important examination and evaluation method for staging of knee cartilage lesions [17].

With the development of AI, deep neural network algorithm has been applied more and more widely in various fields [18, 19]. Some researchers have studied and analyzed the application of BP neural network in medical ultrasound image denoising. The results showed that the BP neural network has a good denoising effect on the ultrasonic image and can also preserve the edge features of the ultrasonic image well [20]. Other researchers studied the feed forward neural network ultrasonic diagnosis method based on BP algorithm and proposed the results of continuous clinical testing. BP neural network ultrasonic diagnosis software can not only improve the efficiency of ultrasonic diagnosis and reduce the time of medical treatment but also use expert knowledge base to share expert knowledge, so as to improve the accuracy of disease diagnosis [21]. The BP neural network algorithm in AI algorithm was used to process the ultrasonic image of knee cartilage to study the stage of cartilage lesions, and a good effect was obtained. The adoption of BP neural network algorithm is very wide, not only in the medical field. For example, some research experts have done a study on using the denoising characteristics of the BP neural network to deal with the noise in seismic data. The experimental results showed that if BP neural network was used to denoise the seismic data, the peak signal-to-noise ratio was greatly improved, and the details of the effective information were well protected, which was in line with the expected results [22]. For the evacuation of public places, the simulation of subway station building based on the deep neural network model is used to conduct evacuation training.

## 5. Conclusion

In this study, it observed the cartilage degeneration stage of KOA under arthroscopy as the standard, observed the consistency between the ultrasound images of KOA cartilage lesions processed by the BP neural network algorithm and the conventional ultrasound images and the results under arthroscopy, and compared the results of the two groups. The results showed that the inspection effect of the ultrasonic image processed by the BP neural network was better than that of the conventional ultrasonic image. However, due to the small amount of data in this study, there was a lack of strong representativeness, but it also reflected the good application prospect of neural network technology in image processing. In the future, more ultrasound images will be optimized to improve the recognition accuracy of the neural network and bring more convenience for clinical ultrasound image diagnosis.

## Figures and Tables

**Figure 1:** KOA diagnostic criteria customized by the American Association of Rheumatology (ACR) in 2001.

**Figure 2:** Process of high-frequency ultrasound examination.

**Figure 3:** Comparison of ultrasound images (a) before and (b) after BP neural network algorithm processing. The red arrow refers to the articular cavity.

**Figure 4:** The manifestations of different stages under arthroscopy. (a) Stage I. (b) Stage II. (c) Stage III. (d) Stage IV.

**Figure 5:** The ultrasound imaging manifestations of different stages in the control group. (a) Normal. (b) Stage I. (c) Stage II. (d) Stage III. (e) Stage IV.

**Figure 6:** The ultrasound imaging manifestations of different stages in the experimental group. (a) Normal. (b) Stage I. (c) Stage II. (d) Stage III. (e) Stage IV.

**Figure 7:** Comparison of the staging results of the two groups of ultrasound images with the results under arthroscopy. A: staging accuracy. B: kappa coefficient. ^*∗*^: the kappa value of the two groups was statistically significant (*P* < 0.05).

**Table 1:** Staging criteria of knee cartilage degeneration under arthroscopy.

Stage	The state of cartilage lesions
Stage I	The cartilage tissue loses its luster and becomes hard in texture
Stage II	The surface of the cartilage is not smooth, with blisters or velvet-like changes, and the invasion range of the damage is less than 1/2 of the depth of the cartilage.
Stage III	The cartilage lesions are severe, with local thinning or even fibrosis, and the invasion range of the injury is more than 1/2 of the cartilage depth.
Stage IV	The cartilage has ulcerated lesions, complete defects, and exposed subchondral bone tissue.

**Table 2:** Staging criteria of knee cartilage degeneration under ultrasound detection.

Stage	Cartilage status under ultrasound
No lesion	The surface shows high echo and the lines are smooth, clear, and continuous. The boundary between cartilage and its inferior bone is normal, and the lower vocal cords are evenly distributed and of normal thickness.
Stage I	The change degree is small or the surface is rough, the thickness is close to normal, the degenerated deep layer shows high echo, the sound line is continuous, the smooth slightly less, and the internal echo distribution is basically uniform
Stage II	The surface shows hyperecho and coarse sound line with localized uplift. The deep sound line of the lesion site shows continuous hyperecho with increased echo and uneven distribution.
Stage III	Thin, with obvious defect, but no invasion of subchondral tissue, uneven distribution of low vocal cords, cartilage interruption defect, degenerative deep high echo, irregular voice line increase, showing extremely coarse, local defect
Stage IV	The subchondral bone is exposed, the deep high echo line is discontinuous, the central low echo cord is thinned, the cartilage defect area is enlarged, and the subchondral bone is invaded, obviously thinned, and the whole layer is thinned.

**Table 3:** Staging results of different articular surface cartilage lesions under arthroscopic examination (place).

Staging		Inspection area				
		Stage I	Stage II	Stage III	Stage IV	Total
Central groove of pulley	The central sulcus	10	18	11	7	164
	The inside of the slope	12	18	16	17	
	The outside of the slope	9	17	18	11	

The femoral	The medial condyle	12	21	25	27	155
	The lateral condyle	12	11	24	23	

**Table 4:** Results of different articular surface cartilage lesion stages in the control group (place).

Staging		Inspection area				
		Stage I	Stage II	Stage III	Stage IV	Total
Central groove of pulley	The central sulcus	7	11	10	11	164
	The inside of the slope	6	20	17	26	
	The outside of the slope	5	17	20	14	

The femoral	The medial condyle	15	22	25	5	120
	The lateral condyle	7	29	11	8	

**Table 5:** Results of different articular surface cartilage lesion stages in the experimental group (place).

Staging		Inspection area				
		Stage I	Stage II	Stage III	Stage IV	Total
Central groove of pulley	The central sulcus	8	16	11	9	169
	The inside of the slope	7	20	18	25	
	The outside of the slope	7	15	20	13	

The femoral	The medial condyle	13	20	20	22	138
	The lateral condyle	9	16	18	20	

## Data Availability

The data used to support the findings of this study are available from the corresponding author upon request.
